The article "Recurrent Neural Networks for Feature Extraction from Dengue Fever" was retracted in 2023. Reasons: signs of a paper mill; suspected computer-generated content; unreliable results or conclusions; concerns about the data.

# Recurrent Neural Networks for Feature Extraction from Dengue Fever

**DOI:** 10.1155/2022/5669580

**Published:** 2022-06-09

**Authors:** Jackson Daniel, S. Irin Sherly, Veeralakshmi Ponnuramu, Devesh Pratap Singh, S. N. Netra, Wadi B. Alonazi, Khalid M. A. Almutairi, K. S. A. Priyan, Yared Abera

**Affiliations:** ^1^Department of Electronics and Instrumentation Engineering, National Engineering College, Kovilpatti, Nallatinputhur, Tamil Nadu 628503, India; ^2^Department of Information Technology, Panimalar Institute of Technology, Chennai, Tamil Nadu 600123, India; ^3^Department of Computer Science and Engineering, Saveetha School of Engineering, Saveetha Institute of Medical and Technical Sciences, Chennai, Tamil Nadu 600124, India; ^4^Department of Computer Science and Engineering, Graphic Era Deemed to be University, Dehradun, Uttarakhand 248002, India; ^5^Department of Information Science and Engineering, East Point College of Engineering and Technology, Bengaluru, Karnataka 560049, India; ^6^Health Administration Department, College of Business Administration, King Saud University, P. O. Box: 71115, Riyadh 11587, Saudi Arabia; ^7^Department of Community Health Sciences, College of Applied Medical Sciences, King Saud University, P. O. Box: 10219, Riyadh 11433, Saudi Arabia; ^8^Department of Biotechnology, School of Health Sciences, Faculty of Biology, Medicine and Health, University of Manchester, Manchester, UK; ^9^Department of Technology and Informatics, Ambo University, Woliso Campus, Ambo, Ethiopia

## Abstract

Dengue fever modelling in endemic locations is critical to reducing outbreaks and improving vector-borne illness control. Early projections of dengue are a crucial tool for disease control because of the unavailability of treatments and universal vaccination. Neural networks have made significant contributions to public health in a variety of ways. In this paper, we develop a deep learning modelling using random forest (RF) that helps extract the features of the dengue fever from the text datasets. The proposed modelling involves the data collection, preprocessing of the input texts, and feature extraction. The extracted features are studied to test how well the feature extraction using RF is effective on dengue datasets. The simulation result shows that the proposed method achieves higher degree of accuracy that offers an improvement of more than 12% than the existing methods in extracting the features from the input datasets than the other feature extraction methods. Further, the study reduces the errors associated with feature extraction that is 10% lesser than the other existing methods, and this shows the efficacy of the model.

The article "Recurrent Neural Networks for Feature Extraction from Dengue Fever" was retracted in 2023. Reasons: signs of a paper mill; suspected computer-generated content; unreliable results or conclusions; concerns about the data.

## 1. Introduction

An estimated more than a billion gets affected each year with neglected tropical diseases (NTDs) in 149 countries throughout the tropics and subtropics [1]. These diseases are caused by parasitic, viral, and bacterial parasites, viruses, and bacteria and are transmitted by mosquitoes. Among the most common NTDs types are borne viruses regarded as a virus collection and naturally transmit between the hosts. Although the clinical appearance of these disorders is well known [2, 3], it is difficult to make an appropriate diagnosis of these conditions. In order to make an accurate arboviral diagnosis, a range of factors must be considered, the most prevalent of which are included in the scientific literature. One factor to consider is that arbovirus is typically asymptomatic, meaning that it may be present in a population without creating an outbreak. The second issue is that their illnesses are frequently difficult to distinguish from one another. They all have similar symptoms, which include arthralgia, fever, headache, myalgia, and orbital pain [4], among other things. Although the symptoms of Dengue, Zika, and Chikungunya are distinct from one another [5, 6], all of them, except for Chikungunya, which is associated with joint discomfort, necessitate a high level of clinical competence and understanding in order to be accurately diagnosed.

Because of the vast range of signs and symptoms associated with these illnesses, it may be difficult to diagnose them. Patients who are infected with dengue may not show any symptoms at all, making it difficult to diagnose the virus in these cases. In most cases, a diagnosis of dengue is confirmed seven to ten days after a mosquito bite [7]. Some of the individuals tend to experience certain symptoms like headache, fever, muscle and joint soreness, and fatigue. Because of the disease progression, some individuals experience organ damage, bleeding, and leakage of plasma [8]. It is possible to divide dengue into the feverish and critical stage. The fever symptoms last between two and seven days. The dengue critical phase, which lasts 24–48 hours and begins with defervescence, is the most dangerous phase of the disease. Severe dengue symptoms, such as plasma leakage or fluid accumulation, as well as respiratory problems, serious bleeding, or organ malfunction, can result in death [9]. A Chikungunya infection can induce symptoms like those of dengue fever, but with more severe joint pain and swelling. The development of Chikungunya is divided into three stages.

Rheumatoid arthritis is characterized by a high temperature, a rash, and discomfort in both the small and large joints, among other symptoms (RA). Throughout the subacute phase, the arthralgia gets worse. Despite the low fatality rate associated with the Chikungunya virus, it has the potential to become chronic [10]. Many people suffer from post-Chikungunya rheumatism, which can last for several weeks or even years and has a detrimental influence on their overall quality of life. Among the symptoms of Zika infection, the most serious is congenital Zika syndrome (CZS). When it comes to pregnancy, there is always a risk of infection [11].

The article "Recurrent Neural Networks for Feature Extraction from Dengue Fever" was retracted in 2023. Reasons: signs of a paper mill; suspected computer-generated content; unreliable results or conclusions; concerns about the data.

When arbovirus infections are detected early, they have the potential to have a substantial impact on a patient's clinical course and therapy and care options. Inadequate arbovirus diagnosis is exacerbated by competing demands for finances and competent and experienced people, due to the presence of multiple disease epidemics at the same time. The development of low-cost, novel, and scalable solutions for the epidemiological surveillance of diseases is urgently required. For example, one strategy is the building of computational models using symptoms and clinical data for the purposes of monitoring and diagnostic classification.

ML/DL models (Figure 1 is frequently developed in field of biotechnology for improving the disease prediction and diagnosis. The models include both training and developmental models, where the training models involve artificial intelligence, machine learning, and deep learning. AI is considered as a computer science discipline that makes predictions based on prior experiences by analyzing data and patterns. The quality and quantity of data are crucial for the learning process to be successful and, as a result, for the accuracy of model predictions to be guaranteed. Finding the optimal combination of parameters that results in a model that can generalize and perform satisfactorily when confronted with previously unknown new data is the key to designing a machine-learning model.

DL is a subfield of machine learning that focuses on learning by layering on successively more meaningful representations and is a subfield of artificial intelligence. DL is a subfield of mathematical logic. When used in this context, the term deep alludes to the concept of piling up representations on top of one another in layers.

According to the latest research, models based on early neural network (NN) iterations are gradually becoming the most effective machine learning (ML) technique (Figure 2) due to their capacity to combine feature extraction and categorization at the same time. The ML models in specific involves supervised and unsupervised modelling, where the supervised models operate mainly on classification and regression tasks. The unsupervised models involve clustering and dimensionality reduction techniques. When it comes to the health sector, the fact that most DL models operate as black boxes presents a significant problem because the industry values openness and accountability. As a result, interpretable machine learning models are becoming increasingly common.

The article "Recurrent Neural Networks for Feature Extraction from Dengue Fever" was retracted in 2023. Reasons: signs of a paper mill; suspected computer-generated content; unreliable results or conclusions; concerns about the data.

In this paper, a random forest (RF) deep learning model is utilized to extract dengue illness variables from text datasets using deep learning techniques. The proposed technique for the model includes data collection, input text preprocessing, and feature extraction, all of which are included in the recommended methodology. Dengue datasets are reviewed to see whether the RF feature extraction method is effective. Using a simulation, the RF model is tested against a range of datasets. According to the simulation findings, the proposed strategy is more accurate than the other methods at extracting features from the input datasets compared to the other methods.

## 2. Related Works

In [12], the authors developed decision tree models. It was established that 1,200 data points from individuals suffering from acute febrile illness might be utilized to develop the Dengue Diagnostic Model, which was later refined (DDM). The Dengue Severity Prediction Model (DSPM) was developed with data from 161 patients with the goal of classifying the severity of dengue in adults. It was necessary to make comparisons between Naive Bayes and SVM to establish whether that patient is affected with dengue. In order to find the ideal hyperparameters of SVM, the gamma parameter and the cost parameter were varied in a grid search. Despite the use of the Grid Search, it was not possible to determine the optimal Naive Bayes configuration. Despite having reduced rate of sensitivity, SVM is found to be the most successful (47%) overall. The Naive Bayes model sensitivity is extremely high, as evidenced by its 18% accuracy rate.

In [13], the authors presented an MLP, two decision trees, and a Bayesian network as alternative models (C4.5 as well as CART). It was not possible to find documentation for the model configurations [14]. Among the models examined, the CART model produced the most accurate results, scoring an *n* error on every metric. The hyperparameter optimization and feature selection are not discussed in detail. One possible explanation for these results is that the ML models are found to be overfitting with small number of records in the dataset (20 records).

In [15], the authors offered three ML models to determine the condition of patients with dengue or not using decision tree model, NN model, and Naive Bayes model. The other models, on the other hand, produced findings that were comparable. In their dataset [15], using SVM and decision tree models, researchers were able to determine whether the patient is affected with dengue, according to the findings of the study [16]. There was no precision information supplied on the model configurations. Throughout this investigation, WEKA was utilised to conduct the experiments and generate the metrics. Because of the high-performance outcomes, there is a chance of overfitting.

The article "Recurrent Neural Networks for Feature Extraction from Dengue Fever" was retracted in 2023. Reasons: signs of a paper mill; suspected computer-generated content; unreliable results or conclusions; concerns about the data.

Reference [17] used clinical data to develop classification models for dengue, including a logistic regression, decision tree, and CNN model. Cross-validation tests with a *k* = 10 sample size were effective in validating and testing the models. For feature selection, the crude odds ratio and modified odds ratio analyses were utilized, respectively. When only four criteria were utilized in all the investigations, the AUC was close to 84% in all of them. The CNN fared somewhat better than logistic regression and decision trees compared with the other two methods. Reference [18] developed the decision tree model for the classification of pediatric patients affected with dengue as two classes (severe or nonsevere) based on severity. According to [18], trees 3, 4, and 5 were not included in the study since the study failed to demonstrate significant improvement compared to the control trees.

Reference [19] developed a model using CART decision tree for the severity assessment on Dengue based on laboratory and clinical data collected from patients. The authors used logistic regression to determine the relative importance of each attribute to the overall image. The hematocrit of the patients was the most important predictor of severe dengue. Although the logistic regression was used to select the features, only 65% of the measures evaluated met or exceeded this criterion.

During a study conducted by [20], patients were classified as either high risk or low risk, allowing for the development of a binary categorization of dengue risk. To solve the classification problem, an MLP model and a grid search model for optimizing the configuration using the modification of certain parameters that include neurons, the number of layers, and the number of layers per class (momentum, number of neurons, iterations, and learning rate) were provided. A self-organizing map (SOM) was used to select seven qualities, and the model was accurate to within 70% of the true value.

The decision tree employed by [21] was utilised to categories patients into four groups: DF, DHF1, DHF2, and DHF3. The features that were utilized to construct a decision tree were provided for each experiment, but the attributes of datasets themselves cannot be provided. Dengue was classified into three groups based on their study of eight different categorization models: dengue fever (DF), dengue heart failure (DHF), and dengue syndrome (DSS). The best results were obtained using the NN model in scenario (1), where the accuracy, precision, and sensitivity of the model were all 71.3%; in Scenario (2), these values were 71.5%; in Scenario (3), they were all 72%. As indicated by the findings, the selection of features did, in fact, result in considerable improvements in the outcomes.

The article "Recurrent Neural Networks for Feature Extraction from Dengue Fever" was retracted in 2023. Reasons: signs of a paper mill; suspected computer-generated content; unreliable results or conclusions; concerns about the data.

Reference [22] used random forest, Naive Bayes, and SVM classification methods to determine if a sample was DHF or non-DHF. It is a bad thing that the model configurations are not documented. All the research in our collection was focused on the binary categorization of dengue, with only two studies trying multiclass categorization of the disease. Multiclass categorization studies focused on the different dengue subtypes and the severity of the sickness. As a result of its simplicity, binary classification has gained universal acceptance. In general, multiclass classification models produce inferior results compared with simpler models because of the difficulty of performing and evaluating them. Tree-based learning techniques are frequently utilized for the problems associated with the process of classification with easier implementation, where the datasets of imbalanced type may lead to degraded performance on the ML models.

Thereby, increasing the shortcomings of the tree splitting criterion used to determine classification accuracy. It was discovered that several studies had been harmed by the overfitting of models. Although each of these investigations used the lowest data sets possible, they were unable to do any additional studies because of the lack of detail in their papers.

## 3. Proposed Method

These are the four stages of our method for predicting severe dengue prognosis using machine learning methodologies. The stages are as follows: data acquisition; data preprocessing; feature selection; classification. The entire procedure is depicted in Figure 3.

The information on dengue fever cases was acquired using epidemiological questionnaires completed by patients during their treatment after the study. The date, location, gender, and age of notified incidents of feature selection were all compiled into a single database. Geocoding is accomplished by the usage of Python modules in each confirmed case location or area.

### 3.1. Data Collection

The proper identification and evaluation of all relevant factors is essential to maintain an effective and accurate healthcare system. Personal, environmental, and health factors have been subdivided as part of the intended Comprehensive Plan of Study (CPS). The data collection module is entrusted with acquiring information about these three variables from the physical world through various means.

The article "Recurrent Neural Networks for Feature Extraction from Dengue Fever" was retracted in 2023. Reasons: signs of a paper mill; suspected computer-generated content; unreliable results or conclusions; concerns about the data.

### 3.2. Random Forest

By analysing historical data, random forest (Figure 4, which is a supervised learning technique, can be used to solve problems and predict recurrence. However, it is mostly used in the resolution of problems. The greater the number of trees in a forest, the denser the forest becomes, and this is true for any random forest. Similar methods allow for the extraction of forecasts from arbitrary forests based on information tests using information tests as a basis. In the end, it all boils down to the voting system. Because it averages the findings, this clustering technique exceeds decision trees in terms of performance.

During the training process, random forest generates a range of alternative decision trees that can be used to make decisions. When selecting the mean forecast for regression, the forecasts from all trees are considered, which means that the final expectations are mutual. As a result, it is referred to as an ensemble technique because it draws on a variety of data points to arrive at a single conclusion. The inner workings of the random forest computation.

*Step 1.* The first stage is to select instances from a dataset at random using a computer programme.
*Step 2.* Create an option tree for each situation that you encounter. The projected outcome of each decision tree will then be displayed.
*Step 3.* In this phase, votes will be cast for each predicted outcome that is presented.
*Step 4.* The final stage is to choose the forecast that is the most accurate based on the cast ballots. When using the random forest procedure to deal with relapse problems, make sure to apply MSE to each and every hub of your data.
  (1) $$\begin{array}{c} \text{MSE}=\frac{1}{N}\sum_{i=1}^{N}{\left(f_{i}-y_{i}\right)}^{2}, \end{array}$$
where *N* is the data points, *f*_*i*_ is the value returned by system, and *y*_*i*_ is the actual value for data *i.*

When utilising random forests to group information, you should be aware that the Gini file (the method used to pick the distribution of tree branch hubs) is frequently utilized, so you should be cautious. This equation, which is based on the class and probability, determines the Gini of each node branches and as a result which branch is the most likely to occur. The database stores pi as the total incidence of a class and the number *c* as the total number of modules.

(2) $$\begin{array}{c} \text{Gini}=1-\sum_{i=1}{\left(p_{i}\right)}^{2}. \end{array}$$

To decide which way the hub should branch, entropy considers the probability of a particular occurrence. This record, in contrast to the Gini record, is significantly more numerically inflated because it is calculated using the logarithmic capacity of the population.

(3) $$\begin{array}{c} \text{Entropy}=\sum_{i=1}^{C}-p_{i}*\;\log_{2}\left(p_{i}\right). \end{array}$$

The article "Recurrent Neural Networks for Feature Extraction from Dengue Fever" was retracted in 2023. Reasons: signs of a paper mill; suspected computer-generated content; unreliable results or conclusions; concerns about the data.

### 3.3. Classification

As previously indicated, the scikit-learn library was utilized in the development of the ANN. The logistic sigmoid function was used as the activation function, and the weight optimization was carried out using a BFGS with a restricted amount of memory. Searches in *b*_*i*_-dimensional space (layers × neurons) using stratified *k*-fold cross validation with *k* = 10 gave the optimal topology, which had an initial value of 0.001. The best topology was found by using stratified *k*-fold cross-validation with *k* = 10.

## 4. Results and Discussions

To assess classification performance, two strategies were used: a test-set technique, which used 25 cases that were unknown to the ANN, and a boosted resubstituting method, which used just 100 training samples. It was never necessary to use the test set when building an ANN classifier; instead, the SVM-RFE technique was employed to discover features, which were then used to train the classifier. In this case, because the test set size is small, the boosted error estimator can be used to verify the results of the test set.

Accuracy can be calculated, which displays the number of correctly labelled positive class samples. Precision, on the other hand, is used to determine the number of correctly labelled positive class samples. Rather than this, positive class-recall is used to predict the total number of accurate samples categorized as belonging to the positive class, which is then divided by the total number of samples to arrive at a prediction. The mathematical formula for recall is provided as follows:

(4) $$\begin{array}{c} \text{Accuracy}=\frac{TP+TN}{TP+FP+FN+TN}\times 100,\\ \text{Precision}=\frac{TN}{FP+TN}\times 100,\\ \text{Recall}=\frac{TP}{TP+FN}\times 100,\\ \text{Error Rate}=100-\text{Accuracy}, \end{array}$$

where TP is the true positive, TN is the true negative, FP is the false positive, and FN is the false negative.

Dengue outbreak forecasting on a large scale is generally done to provide an early warning system. The use of finer granularity in intraurban prediction seeks to identify places that will be more vulnerable soon, allowing for more accurate prevention and management despite the lack of available financing. As a result, besides calculating the Pearson correlation coefficient between the anticipated and actual case counts, we developed a hit rate measure to evaluate the forecasting performance from a spatial standpoint, by evaluating the model ability to locate high-risk urban units throughout the town boundaries.

The article "Recurrent Neural Networks for Feature Extraction from Dengue Fever" was retracted in 2023. Reasons: signs of a paper mill; suspected computer-generated content; unreliable results or conclusions; concerns about the data.

In this scenario, having a higher sensitivity is advantageous because SD is an absolute requirement. According to the accuracy metric, the percentage of projected positive cases that occur is calculated as follows. It becomes clear when we compare the proposed technique to the two other methods of error estimation that it has higher precision rates.

Because of the high precision and recall of the proposed method, it obtained a favourable F1 evaluation. Because the number of SD and DF patients in the data set is not fairly distributed over the population, the estimations of accuracy, precision, and F1-score may be skewed because of this. Keeping this in mind will help you when analyzing the information. Because of this, there would be no difference in the outcomes of sensitivity (recall) and specificity (precision), which are independent of the data set or population prevalence.  Figure 5 depicts the accuracy rate.

A comparison of the proposed RF technique with existing NN and SVM classifiers reveals that it outperforms them in terms of overall performance and accuracy. Without the usage of RF technology, all classifiers, including the proposed ANN, performed worse than they would have otherwise. For example, the accuracy of proposed method was 80%, the accuracy of NN was 70%, and the accuracy of SVM was just 78.7% in this experiment. As a result, the samples are validated using nearest neighbours in ANN, whereas the SVM and NN focused on training samples and consumed a considerable amount of data for disease prediction. As a result, RF is used to select the most advantageous characteristics. The proposed method achieved an accuracy of 88% as a result of RF, SVM achieved an accuracy of 80%, and NN achieved an accuracy of 72%, all of which were superior to the baseline. Compared to existing approaches, the accuracy of the new RF with the ANN methodology is much higher. Because, in this experiment, the DWT technique minimised feature deterioration while SVM and NN did not, the DWT technique is recommended. In addition, the proposed RF strategy efficiently selects the relevant feature for the ANN method, which adaptively learns the data for classification using the selected feature.

The accuracy of SVM predictions was only 35% of that of ANN and NN predictions, which were not influenced by the FS method, respectively. This is a statistically significant distinction. Although SVM performed well on both unstructured and semistructured data, it performed badly when the target classes were similar in their characteristics. The NN achieved a precision of 65% in the final forecast without the use of the RF algorithm, but this increased by around 3% when the RF approach was utilised. A model requires more than thousands of data points to be trained, which is why it is so expensive to build. Because only a small amount of data is used in the research for the prediction of muscular paralysis conditions, artificial neural networks (ANNs) are used, and RF methods were used to achieve 85%.

The article "Recurrent Neural Networks for Feature Extraction from Dengue Fever" was retracted in 2023. Reasons: signs of a paper mill; suspected computer-generated content; unreliable results or conclusions; concerns about the data.

The ANN approach has several advantages, two of which are instance-based learning and adaptive learning for categorization. However, the greater the number of elements in a system is, the less effective the system is at final classification. This has resulted in the development of RF, which has achieved an accuracy rate of 88% when using an ANN. The recall value of the proposed RF using the ANN approach is depicted in Figure 6.

The results of the analysis show that the RF approach outperforms the standard classifier in terms of recall value. The ANN achieved only about 75% to 78% of recall values for both the FS and the SVM/ANN techniques, compared with 75% to 77% for the other two approaches. While not employing perfect features for the prediction process of muscular paralysis, the SVM gets 83% recall values when using the FS methodology. However, the same technique reduces its performance to 2% when using the FS methodology. When combined with artificial neural networks, the proposed RF technique extracted the relevant properties from the signal with an 81% recall value. With too many features comes poor performance, so the RF algorithm was used to choose the most suitable characteristics, which when combined with ANN technology, resulted in a recall value of 89%. ANNs have the advantage of being able to learn from data and categorise it in an adaptable fashion, which is a significant advantage. The comparison between the proposed RF with the ANN approach and the NN and SVM methods is shown in Figure 7.

According to our evaluation results, the proposed RF technique using ANN exhibits a lower error rate than neural networks and support vector machines. While all other approaches have lower error rates, NN has the highest, with a 0.28% error rate without FS and a 1% error rate reduction combined with RF. The high error rate of NN can be attributed to the fact that it requires a considerable amount of training data although only a small number of samples were employed in this experiment. The current SVM has an error rate of 0.18 to 0.19, both with and without FS, and exceeds NN in terms of performance despite these disadvantages. When only the RF feature extraction technique is used, the proposed ANN has an error rate of 0.19, which is quite good. Because of the need for a lower error rate, only the relevant signal features were retrieved by the proposed FE technique to achieve that goal.

The article "Recurrent Neural Networks for Feature Extraction from Dengue Fever" was retracted in 2023. Reasons: signs of a paper mill; suspected computer-generated content; unreliable results or conclusions; concerns about the data.

The system warns key stakeholders of potential health hazards and dispatches medical help as soon as a dengue outbreak is detected, based on a real-time risk assessment based on infection and cardiovascular disease (CVD) risk levels. It is intended that the proposed system, which operates in a cloud environment, will protect user sensitive information from being exposed and identify the critical locations and users who are responsible for virus transmission. All components of diagnosis, monitoring, and risk depiction are organised in the intelligent healthcare system that has been proposed.

The efficiency evaluation of the various components of the proposed system justifies the use of the system under consideration. Additionally, the RF-based health risk classification surpasses the alternatives in terms of statistical performance, and this is confirmed by evaluations of the preprocessing and its performance, in addition to the alert generation and RF outbreak risk assessment performed. Although this method is now only applicable to the heart, it has the potential to be expanded to include other vital organs in the future, such as infection and other illnesses that impact these organs.

## 5. Conclusions

In this paper, the RF for the model includes data collection, input text preprocessing, and feature extraction, all of which are included in the recommended methodology. Using dengue datasets, it is investigated if RF-based feature extraction is effective at extracting features from the datasets. In a simulation, the RF model is evaluated against a variety of different datasets. According to the simulation findings, the proposed strategy is more accurate than the other methods at extracting features from the input datasets compared to the other methods. Although both neural networks and SVM are traditional classifiers, the research shows that the newly presented approach surpasses both. When using the RF approach, the ANN achieved 88% accuracy and 89.9% recall, but the NN achieved 72% accuracy, 77% recall, and a 0.27 error rate when used in conjunction with the RF method. However, only 80% of the proposed ANN was accurate, while 75% of the current NN was accurate, and 75% of the current NN was implemented with the Relief-F technique, resulting in an error rate of 0.195. Based on this data, it can be concluded that FS has a major role in the prediction of muscle paralysis in the elderly. Future studies on the methodology will include the use of deep learning multiscale strategy for the prediction of a wide range of diseases in the future. Further, the methods on neural network can be studied to avoid the problem of overfitting due to the inputs from the previous layers.

The article "Recurrent Neural Networks for Feature Extraction from Dengue Fever" was retracted in 2023. Reasons: signs of a paper mill; suspected computer-generated content; unreliable results or conclusions; concerns about the data.

## Figures and Tables

**Figure 1:** ML/DL model.

**Figure 2:** Machine learning techniques.

**Figure 3:** Proposed model.

**Figure 4:** Random forest model [23].

**Figure 5:** Accuracy rate.

**Figure 6:** Precision rate.

**Figure 7:** Recall rate.

## Data Availability

The data used to support the findings of this study are included within the article. Further data or information is available from the corresponding author upon request.
